# Inactivation of tumor suppressor gene pten in early and advanced gallbladder cancer

**DOI:** 10.1186/s13000-015-0381-2

**Published:** 2015-08-21

**Authors:** Iván Roa, Gonzalo de Toro, Fernanda Fernández, Anakaren Game, Sergio Muñoz, Xabier de Aretxabala, Milind Javle

**Affiliations:** Creative Bioscience Santiago, Avenida Del Valle Norte 857. Oficina 102, Ciudad Empresarial, Huechuraba Santiago, 8580702 Chile; Servicio de Anatomía Patológica Hospital de Puerto Montt, Puerto Montt, Chile; Centro Diagnóstico Histopatologia-Citopatologia, Temuco, Chile; Facultad de Medicina, Universidad del Desarrollo, Santiago, Chile; Departamento de Salud Pública, CIGES, Facultad de Medicina, Universidad de la Frontera, Temuco, Chile; Departamento de Cirugía, Clínica Alemana, Santiago, Chile; Javle, Milind UT-MD Anderson Cancer Center, Houston, TX USA

## Abstract

**Background:**

PTEN is a tumor suppressor gene that regulates the PTEN/PI3k/AKT/mTOR pathway, which is frequently altered in human cancers including gallbladder cancer (GBC). To determine the frequency of PTEN expression in GBC and to establish its relation to clinical and morphological parameters and survival in GBC.

**Methods:**

The immunohistochemical expression of PTEN was studied in 108 GBC. All the cases included areas of non-tumor mucosa adjacent to the tumor.

**Results:**

The group was comprised of 108 patients, 91 women (84.3 %) and 17 men (15.7 %) with an average age of 65.2 years (SD ± 12.3 years). Thirty-five cases (33 %) were early carcinomas (EC) and the remaining 73 (67 %) were advanced cases (AC). All the internal controls were positive (moderate or intense in 96.3 %). Only in three AC (4.1 %) was there a complete absence of PTEN immunohistochemical expression. There were no significant differences in relation between PTEN expression and tumor infiltration or degree of differentiation. The three patients with PTEN inactivation died before 10 months; however, the other patients with AC had a survival of 53 % at 10 months.

**Discussion:**

Loss of PTEN expression was observed in 4.1 % of the advanced GBC. All the patients with this alteration died before 10 months. PTEN inactivation could be a rare event, but with a poor prognosis in advanced GBC.

## Background

For many years Chile has had the highest incidence and mortality due to GBC in the world, in both genders, and it represents the second cause of death by malignant tumors in women in Chile [1–3]. Other Indo-American countries like Bolivia, Mexico and Ecuador follow in frequency, and in Asia countries such as India and Pakistan [2, 4]. GBC ranks 20th among all malignant tumors with an incidence of 2.2 × 10^6^ inhabitants, and 22nd for mortality (0.7 × 10^6^) with a prevalence at 5 years of 16.8 × 10^6^ inhabitants [2].

As with other epithelial malignant tumors, GBC is the result of multiple genetic alterations involving multiple genes from different metabolic pathways, the importance of which has not yet been clearly established [5–9]. Numerous somatic mutations have been reported for GBC, of which only a small subgroup contributes to tumor progression. The distinction has been made only recently between mutations in the “driver” or controller genes of the multiple mutations in neutral or “passenger” genes that contribute in only a small way to cancer development [10, 11]. The most frequently mutated genes in GBC are TP53 (47.1 %), KRAS (7.8 %) and ERBB3 (11.8 %) (https://www.sanger.ac.uk/). It has also been shown recently that the signaling pathway of ErbB, which includes EGFR, ERBB2, ERBB3 and ERBB4, is one of the most frequently altered in GBC [12, 13].

PTEN (phosphatase and tensin homolog) is a tumor suppressor gene located on chromosome 10q23. 3. PTEN encodes a protein with a phosphatase function which, as it removes phosphate groups, inactivates substrates and thus acts as a tumor suppressor gene [9, 14]. The functional loss of PTEN may be the result of somatic mutations, deletion or inactivation (LOH, methylation), abnormalities in transcriptional and post-transcriptional regulation, microRNAs, regulation of microRNAs, or due to alterations in the mechanisms that regulate the stability and degradation of the PTEN protein [15, 16]. The absence of the functional protein PTEN enables unfettered PI3k activity, which determines the uncontrolled production of PIP3, one of the most important effectors of the PI3K/AKT pathway, with mTOR stimulating protein synthesis and initiating onset of the G1 phase of the cell cycle and interacting with proteins that regulate apoptosis [17].

Germline loss of PTEN is the hallmark of Cowden syndrome [18], while sporadic alterations in PTEN have been observed in a broad spectrum of malignancies [19]. The multiple mechanisms that lead to PTEN inactivation render their study difficult; therefore, determining a gene’s protein expression is considered a good way to assess the functional status of the gene [20–22]. The absence of expression is considered a reflection of inactivation of the gene, independent of its cause.

The aim of this work was to determine the distribution and inactivation frequency of PTEN in EC and AC of GBC and to establish the correlation with clinical and morphological parameters and survival. An additional aim was to consider indirectly the importance that PTEN inactivation may have in the deregulation of the PI3K/AKT pathway in GBC.

## Methods

### Cases and controls

108 cases of primary gallbladder adenocarcinomas diagnosed in the Puerto Montt Regional Hospital and the Temuco Diagnostic Center were included. In each case, a representative inclusion of the tumor was selected (anonymized archive material of formalin-fixed, paraffin-embedded tissues). In all 108 cases, areas of non-tumor mucosa adjacent to the neoplastic lesions were used as an internal control. This work was approved by the Ethics Committee of the National Fund for Scientific and Technological Development (FONDECYT) and that of the Faculty of Medicine of the Clínica Alemana-Universidad del Desarrollo.

### Immunohistochemical technique

The immunohistochemical study was performed on complete histological sections, taking the lack of information regarding the degree of heterogeneity of PTEN protein expression in this and other neoplasias into consideration. The standard automated immunohistochemical technique for fixing tissue in formalin and embedding it in paraffin was used. The 4-micron thick histological sections were deparraffinized and hydrated in decreasing alcohol concentrations. Antigens were recovered by exposure to microwaves in citrate buffer pH 6.0 and washed in PBS pH 7.4. The monoclonal antibody PTEN (D4.3) (XP® Rabbit mAb Cell Signaling) was used in a dilution of 1:125. The primary antibody was incubated at room temperature for 60 min and then incubated with the complex Super Picture Polymer Detection Kit™ Zymed in a Dakoautostainer™. All determinations were made in a single run to avoid variations in the assessment conditions.

### Methods for measuring positivity

The immunohistochemical positivity was expressed by means of cytoplasmic and nuclear staining with slight membrane reinforcement in both the normal and tumor cells. Positivity was estimated according to the following scale used by other authors [22]: intensity 0 = (negative), 1 + (weak), 2+ (moderate or intense). Positivity percentage = 0 % (negative), > 1–100 % (positive). All the cases included areas of non-tumor tissue. Positive staining was measured based on a comparison between the non-tumor mucosa and the tumor. Tests were also performed with homologous scales that included factors like staining intensity and an estimation of the percentage of positive cells [21]. The score obtained enabled an ROC analysis to determine the greatest degree of sensitivity and specificity of the immunohistochemical staining [23]. However, there were no significant differences in terms of the semi-quantitative estimation initially described.

### Sample determination

Given the limited available information regarding PTEN/PI3K/AKT/mTOR alterations in GBC, an estimate was made based on previous reports in other malignancies. For most of the markers used, there is very little information regarding patient survival. It was expected that a 20 % mutation frequency and altered immunohistochemical protein expression between 5 and 50 % of the cases would be observed. Greater positivity was expected in locally advanced tumors. In the control group (non-tumor), it was expected that positivity of mutations or abnormal expression would be found in less than 3 and 10 % of the cases, respectively. As an internal control, adjacent non-tumor mucosa were included in all cases where possible. The minimum sample size for analysis was based on the number of predictors. In this study, the markers were considered as each requiring at least ten observations for analysis. The latter estimation provided a final sample size of around 70 patients evenly distributed. For a 95 % confidence interval with a corrected statistical power of 95 %, a minimum of 70 cases and 50 controls were required.

### Statistical analysis

This was done by means of a chi-squared test and Fisher’s exact test for the contingency tables (*p* < 0.05) as well as an analysis of variance for the averages and Kaplan-Meier actuarial survival curves with a log-rank test of significance.

## Results

The group comprised 108 cases, the general characteristics of which are summarized in Table 1. Eighty-four percent of the cases were women with an average age of 65.1 years (SD ± 11.6 years) and the remaining 17 were men with an average of age of 66.1 years (SD ±10.1 years). All the cases were adenocarcinomas. Thirty-five cases (33 %) were EC (17 mucous carcinomas and 18 muscular carcinomas) and 73 (67 %) were AC (29 subserosal carcinomas, 24 serosal, and 20 cases beyond the serosa). The difference in the average ages between the early and advanced carcinomas, as well as the relation between the level of tumor infiltration of the wall and the progression in the average ages was significant (*p* < 0.001). 30.3 % of the tumors were well differentiated, with the great majority being moderately differentiated (51.5 %) or poorly differentiated (18.2 %).

**Table 1:** General features of gallbladder cancer patients

Age	Number	Year	SD
Female	91 (84.3 %)	65.1	±11.6
Male	17 (15.7 %)	66.1	±10.1
Total	108	65.2	±12.3
	*Mínimum 39 years*	*Maximal 90 years*	
Tumor localization	Number	%	
Fundus	25	24.5	
Body	21	17.2	
Neck	7	6.2	
Difusse	13	13.3	
Unnaparent	42	38.8	
	108	100.0	
Histological Type			
Adenocarcinoma	108	100	
Differentiation			
Well	33	30.3	
Moderate	56	51.5	
Poor	20	18.2	
	108	100	
Infiltración level			
Mucosa	17	16	
Muscular	18	17	
Subserosal	29	26.6	
Serosal	24	22.3	
Beyond serosa	20	18.1	
	108	100	

The immunohistochemical staining in the 108 tumors and their respective internal controls are summarized in Table 2. In 96.3 % (104 cases) the non-tumor mucosa showed moderate or intense positivity (2+) and only 3.7 % (4 cases) were weak positive (1+). No negative cases were observed in this group. In the GBC, however, three cases (2.8 %) had an absence of expression or inactivation of PTEN (in the presence of positive internal controls) (Fig. 1). All the cases without PTEN expression were AC, all women (50, 56 and 62 years respectively), one subserosal and two serosal with survival of 3, 6.2 and 9.9 months respectively after diagnosis. The inactivation frequency in the AC patient group reached 4.1 % (3 of 73 cases). Unlike what was observed in non-tumor tissues, the adenocarcinomas had a similar proportion of positivity (1+) or weak compared to a moderate or intense positivity (2+), which could suggest a partial or incomplete degree of PTEN activity.

**Table 2:** Intensity of immunohistochemical expression of PTEN in non-tumor gallbladder mucosa and gallbladder cancer

	Non-tumor mucosa		Gallbladder cancer	
Intensity	Number	Percent	Number	Percent
0	0	0	3	2,8
1	4	3,7	59	54,6
2	104	96,3	46	42,6
	108	100	108	100

**Fig. 1:** PTEN immunohistochemistry expression. **a** Strong cytoplasmic positive expression of PTEN in gallbladder adenocarcinoma. **b** Infiltrating adenocarcinoma with negative PTEN expression in tumor cells and stromal and vascular positivity

Actuarial survival of the group was 41 % at 5 years of follow-up. In the 73 patients with AC, the actuarial survival at 10 months of follow-up was 52 and 29 % at 5 years. However, the three patients who presented immunohistochemical inactivation of PTEN died before the 10 months. Although the number is small and does not permit a statistically valid conclusion, this fact is noteworthy (Fig. 2).

**Fig. 2:** Survival and risk of death. Actuarial survival (*left*) and risk of death (*right*) curves in patients with advanced gallbladder cancer in relation to the absence of expression of PTEN. The three patients with PTEN inactivation died prematurely compared to the advanced cancer patients

## Discussion

Our results show immunohistochemical expression of PTEN protein in all the cases used as internal controls, with this expression being moderate or intense from the immunohistochemical point of view in 96.3 % of the cases, which may reflect normal activity in this gene. No negative cases were observed, which may suggest some degree of PTEN inactivation in the non-tumor mucosa adjacent to the tumors. However, in the GBC there was a greater dispersion in the intensity of the positive staining, being weak in 54.5 % of the cases and moderate in 42.6 %, which may mean that the tumor tissues present a variable expression, possibly a reflection of differing degrees of PTEN activity or inactivation. This being a recessive gene, inactivation of an allele does not necessarily compromise its function entirely, as it can express itself partially [24]. In most tumors the loss of PTEN is monoallelic (gliomas, breast, colon, lung), with biallelic being less frequent [24–27], as inactivation due to methylation of promoter areas is one of the inactivation mechanisms that occurs more frequently than genomic alterations [24, 28, 29]. Thus, the absence of PTEN expression in three cases of advanced GBC suggests is an infrequent phenomenon (4.1 % of all AC) and is also delayed since its inactivation could not be demonstrated through the loss of its expression in any of the 35 EC. There is little information about the inactivation of this gene in GBC measured using different molecular techniques. Some indicate inactivation frequencies ranging between 0 and 5 %, but this does not rule out that other PTEN inactivation mechanisms may be at work [16]. On the other hand, the poor prognosis of the three patients with an absence of PTEN protein expression compared to patients at similar stages must be pointed out [30]. In these patients, PTEN inactivation may have released the PI3k/AKT pathway, which through some of its effectors like mTOR is able to activate cell proliferation [31]. Although PTEN inactivation is observed in around 4 % of the advanced cancers, it is worthy of note that the other inactivation mechanisms in this proliferative pathway and which promote tumor growth and development have recently been reported in significant percentages (http://cancer.sanger.ac.uk, [32–34]), which will open up important expectations for the use of selective blockers and inhibitors of this pathway as a targeted therapy in patients with advanced gallbladder cancers [35–37]. Our recent work has shown activating mutations in exons 9 and 20 of the PI3k gene in 16.9 % of GBC, suggesting that this gene together with PTEN could be a therapeutic target in around 20 % of advanced gallbladder cancers (Roa et al., observations not published).
